RETRACTED

# LncRNA TUG1 promoted KIAA1199 expression via miR-600 to accelerate cell metastasis and epithelial-mesenchymal transition in colorectal cancer

**DOI:** 10.1186/s13046-018-0771-x

**Published:** 2018-05-18

**Authors:** Junfeng Sun, Jiyi Hu, Guojun Wang, Zhen Yang, Chunlin Zhao, Xiefu Zhang, Jiaxiang Wang

**Affiliations:** 1 Department of Gastrointestinal Surgery, The First Affiliated Hospital of Zhengzhou University, No.1 Jianshe East, Zhengzhou, 450052 China; 2 Colorectal Cancer Center, Fudan University, Shanghai, China; 3 Pediatric Surgery, The First Affiliated Hospital of Zhengzhou University, Zhengzhou, China

**Keywords:** lncRNA TUG1, KIAA1199, miR-600, Colorectal cancer, EMT, Metastasis

## Abstract

**Background:**

LncRNA TUG1 has been reported to be highly expressed in CRC samples and cells and promoted metastasis by affecting EMT, indicating a poor prognosis for colorectal cancer (CRC). In this study, we determined the underlying mechanism for tumor oncogenesis of lncRNA TUG1 in CRC metastasis.

**Methods:**

The expressions of miR-600 and KIAA1199 in 76 CRC patients and CRC cells and CRC metastatic tissues were determined using qRT-PCR. Epithelial-mesenchymal transition (EMT)-related proteins were determined using western blot. CRC cell metastasis was assessed by colony formation, wound healing and transwell assay. Luciferase reporter gene assay was used to confirm miR-600 binding to KIAA1199 3’UTR.

**Results:**

Our data showed that lncRNA TUG1 was upregulated in CRC cells, miR-600 was downregulated in CRC tissues, cell lines and CRC metastatic tissues, and low miR-600 expression predicted a poor clinical prognosis. Overexpression of miR-600 suppressed CRC cell migration/invasion and EMT-related proteins in vitro, inhibited tumor volume and weight, and decreased the number of CRC liver metastasis in vivo. KIAA1199 was upregulated in CRC tissues, and was negatively regulated by miR-600. KIAA1199 overexpression promoted CRC cell migration and invasion, which reversed the inhibition effect of miR-600 mimic on migration and invasion of CRC cells. Moreover, TUG1 negatively regulated miR-600, and inhibition of TUG1 suppressed CRC cell migration and invasion and EMT-related proteins via regulating miR-600.

**Conclusion:**

Our study proved that TUG1 promoted KIAA1199 expression to accelerate EMT and metastasis of CRC cell through inhibition of miR-600 expression.

## Background

Colorectal cancer (CRC) is the third most deadly cancer in the United States, which accounts for 8% of all cancer deaths in men and women [1]. It has been estimated that there are nearly 140,250 new CRC cases and 50,630 deaths of CRC in the United States in 2018 [1]. Surgery combined with adjuvant therapy resected cancerous lesions, inhibited CRC cell growth and decreased CRC metastasis{Acciuffi, 2018 #35}, thus reduced the occurance of CRC. However, 40–50% of CRC patients still had metastasis to lymph node, liver, lung, etc. [2–4]. Increasing evidences show that epithelial-mesenchymal transition (EMT) plays an important role in the metastasis of CRC. Li et al. reported that inhibition of EMT induced the suppression of CRC cell migration and invasion [5]. Vu and Datta reviewed that EMT led to the increase of invasiveness and metastasis in CRC [6]. Besides, during EMT, epithelial marker E-cadherin is downregulated, and mesenchymal markers vimentin and N-cadherin are upregulated through regulating different EMT-related signaling pathways [7].

RETRACTED

*KIAA1199* is a gene firstly reported in Deiters’ cells and considered as the cause of non-syndromic hearing loss in 2003. Studies have shown that KIAA1199 was upregulated in many human cancers and negatively related with the survival rate [8, 9]. Researchers have shown that protein level of KIAA1199 was remarkably increased in colon cancer tissues and cells, and indicated markedly reduced survival [10, 11]. KIAA1199, as a cell-migration inducing protein, is overexpressed in metastatic CRC tissue, and inhibition of KIAA1199 inhibited migration and invasion of CRC cells and suppressed CRC metastasis [12]. However, the underlying mechanism of KIAA1199 in CRC is not fully revealed.

microRNAs, a class of small noncoding RNAs that modulate gene expression at post-transcriptional level, are involved in the development, progression and metastasis of CRC cancer [13, 14]. miR-600 was first identified in breast cancer stem cells that regulated the balance between self-renewal and differentiation of breast cancer stem cells and influenced tumor progression [15]. Later, studies showed that miR-600 was downregulated in cancers, such as acute myeloid leukemia, cervical cancer [16, 17], which was associated with a positive prognosis of cancer. Recently, Zhang et al. found that miR-600 overexpression remarkably inhibited migration and invasion abilities of CRC cells [18], however, the underlying mechanism of miR-600 in CRC metastasis is unclear. According to the bioinformatics software Targetscan, there were potential binding sites between miR-600 and KIAA1199. Therefore, we assumed miR-600 as a potential upstream molecular of KIAA1199, and might involve in modulating CRC metastasis.

Researchers have found long noncoding RNAs (lncRNAs) were abnormally expressed in CRC, which was necessary for the proliferation, apoptosis, migration and invasion. Our previous report found that lncRNA TUG1 was upregulated in CRC samples and cells and promoted metastasis by affecting EMT, indicating a poor prognosis for CRC [19]. Bioinformatics software DIANA also predicted there were potential binding sites between TUG1 and miR-600. Thus, we assumed that lncRNA TUG1 promoted KIAA1199 expression via miR-600 to accelerate CRC metastasis and EMT.

RETRACTED

## Methods

### Tissue collection

Seventy-six CRC tissues and matched adjacent normal tissues were collected from CRC patients who received surgical treatment at the department of Gastrointestinal Surgery, the First Affiliated Hospital of Zhengzhou University between March 2016 and June 2017. The patients were divided into two groups: miR-600 high expression group (*n* = 29) and miR-600 low expression group (*n* = 47) according to the mean relative expression level of miR-600 (mean fold 0.55 was used as the cut-off). No patients received radiotherapy, chemotherapy or targeted therapy before surgery. The study was approved by the Ethics Committee of the First Affiliated Hospital of Zhengzhou University, and all patients signed informed consent. All specimens collected from surgery were immediately stored at − 80 °C.

### Cell culture and transfection

Human CRC cell lines (HCT116, SW480, HT29, LOVO and SW620) and the normal human colon epithelial cell line NCM460 were purchased from the American Type Culture Collection (USA). The cells were cultured in Dulbecco’s modified Eagle medium (DMEM) (Gibco, USA) supplemented with 10% fetal bovine serum (FBS) (Gibco, USA) at 37 °C with 5% CO_2_.

miR-600 mimic, miR-600 inhibitor, si-KIAA1199, pcDNA-KIAA1199, si-TUG1 and corresponding scrambled negative control (NC) vectors were synthesized by Invitrogen. Lentivirus miR-600 (lenti-miR-600) and lenti-vector were synthesized by GENECHEM (Shanghai, China). The vectors were transfected into CRC cells by Lipofectamine 2000 (Invitrogen, USA) according to the manufacturer’s instructions.

### Quantitative real-time PCR

Total RNA was extracted from CRC tissues, matched adjacent normal tissues, CRC cells and the normal human colon epithelial cell using Trizol (Invitrogen, USA). cDNA was compounded using the PrimeScript™ RT reagent Kit with gDNA Eraser (Takara, Japan). Real-time PCR was performed to measure miR-600 and KIAA1199 expressions using One Step SYBR® PrimeScript™ PLUS RT-PCR Kit (Takara, Japan). Fold change expression of miR-600 and KIAA1199 was calculated using the 2^−ΔΔCt^ method. Primers used in this study were synthesized by Invitrogen. miR-600 primer 5’-CCCGUCCCGACCGGACUCGUUCCGAGAACAGACAUUCAUUGAGGUGACGGACUGUCUGUUCUCGGAAGGAUACUUCGACCUCGGUGUGUCGUGCACACUGAA-3′; KIAA1199 primer 5’-AGGCGTGACACTGTCTCGGCTACAG-3′.

### Colony formation assay

SW620, LOVO or HCT116 cells were plated in 6-well plates at 1 × 10^3^ cells per well and maintained in DMEM containing 10% FBS for 2 weeks with the medium replaced every 4 days. After 2 weeks, the colonies were washed with PBS for 2 times, fixed with methanol and stained with crystal violet (Sinopharm Chemical Reagent, China). The number of colonies was counted under a microscope.

RETRACTED

### Wound healing assay

SW620, LOVO or HCT116 cells were transfected with miR-600 mimic, si-KIAA1199 pre-NC or si-NC. After 72 h, cells were collected and seeded into 6-well plates until 80% confluence. Then, a pipette tip was used to creat a wound. At 0 and 48 h, the spread extent of wound closure was observed by photograph.

### Transwell assay

SW620 and LOVO cells were transfected with miR-600 mimic or NC, and HCT116 cells were transfected with miR-600 inhibitor. After 72 h, 3 × 10^4^ cells were collected and placed in 100 μl serum-free DMEM medium in the upper chamber coated with Matrigel (BD, USA). DMEM medium supplemented with 10% FBS was added into the lower chamber. Twenty-four hours later, cells that migrated through Matrigel were fixed with methanol and stained with crystal violet (Sinopharm Chemical Reagent, China) for 15 min. To observe the invasion ability, cells were incubated for 48 h. Image J was used to quantify the number of migration and invasion cells.

### Western blot

After transfection, CRC cells were lysed in Radio Immunoprecipitation Assay (RIPA) buffer (Thermo Scientific, USA), and protein concentration was measured by Pierce BCA Protein Assay Kit (Thermo Scientific, USA). Proteins were separated on a 12% SDS-polyacrylamide gel electrophoresis (PAGE) and transferred to polyvinylidene difluoride (PVDF) membrane (Invitrogen, USA), which were blocked with 5% skim milk for 2 h. Blots were incubated with primary antibodies against E-cadherin (Cell Signaling Technology, USA), N-cadherin (Cell Signaling Technology, USA), Vimentin (Cell Signaling Technology, USA), Fibronecin (Abcam, USA), KIAA1199 (Invitrogen, USA), β-actin (Sigma, USA) and horseradish peroxidase-conjugated secondary antibody (Abcam, USA). Protein bands were visualized using ChemiDoc MP imaging system (Bio-Rad, USA). β-actin acted as an internal control.

### Luciferase reporter gene assay

pMIR-KIAA1199 3’UTR Wild Type (WT) (400 ng) or pMIR-KIAA1199 3’UTR mutant (MT) were transfected into HCT116 cells with 40 ng pRL-TK vectors (Promega, USA). miR-600 mimic or miR-600 inhibitor or NC was co-transfected with reporter plasmids for 48 h. Cells were collected to measure luciferase activity by dual Glo™ Luciferase Assay System (Promega).

### Experimental mouse model

BALB/c nude mice (5-week-old, male) were purchased from The Animal Experimental Center of Zhengzhou University, and the animal study was approved by the Ethics Committee of the First Affiliated Hospital of Zhengzhou University. SW620 cells were transfected with lenti-miR-600 or lenti-vector and resuspended at a concentration of 1 × 10^6^ cells//100 μl. A total of 100 μl SW620 cells were subcutaneously injected into each BALB/c nude mouse (*n* = 6). Seven days after inoculation, tumor volume was measured, which was calculated by the formula: 0.5 × length×width^2^. Nude mice were sacrificed after 25 days, and the weight of tumor tissues were measured. In addition, SW620 cells mentioned above were injected into the spleen subcapsular of each BALB/c nude mice at a concentration of 1 × 10^6^ cells/100 μl (*n* = 6) to establish nude mice liver metastasis model of CRC. Nude mice were sacrificed after 5 weeks, and liver tissues were obtained to count tumor nodules.

RETRACTED

### RNA immunoprecipitation (RIP) assay

Magna RIP™ RNA-Binding Protein Immunoprecipitation Kit (Millipore, USA) was used for RIP experiment. Endogenous polycomb repressive complex2 (EZH2) (Invitrogen, USA) was used for RIP assay. Ago2 was assessed by IP-western, and TUG1 and miR-600 levels were measured by qRT-PCR.

### Statistical analysis

SPSS software (version 18.0) was used for data analysis, and the data was expressed as mean ± standard error (SE). The overall survival was calculated using the Kaplan-Meier method. The data was analyzed by one-way ANOVA and t test, with *P* < 0.05 considered statistically significant.

## Results

### LncRNA TUG1,miR-600 expressions in CRC and their effect on CRC cells

Our previous research found lncRNA TUG1 was upregulated in CRC cell lines and CRC clinical samples, and play a vital role in EMT and migration of CRC [19]. Then, we measured the expression of miR-600 in 76 CRC tissue and adjacent normal tissue, and CRC cell lines (HCT116, SW480, HT29, LOVO, SW620) using qRT-PCR. miR-600 expression was decreased in CRC tissues compared with adjacent normal tissues (Fig. 1a). miR-600 expression was significantly decreased in CRC cell lines than the normal human colon epithelial cell line NCM460, with the lowest miR-600 expression in SW620 cell line and the highest in HCT116 cell line (Fig. 1b). In addition, decreased miR-600 expression was found in metastasis CRC tissue compared with the non-metastasis CRC tissue (Fig. 1c). According to the average value of miR-600 expression in CRC patients, we divided the patients into low miR-600 expression group (*n* = 47) and high miR-600 expression group (*n* = 29). Patient characteristics between the low miR-600 and the high miR-600 group were shown in Table 1. Kaplan-Meier curve revealed a poor clinical prognosis for patients with low miR-600 expression (Fig. 1d).

RETRACTED

**Fig. 1:** miR-600 expression was decreased in CRC tissue and cell lines. **a** Seventy-six CRC tissues and matched adjacent normal tissue were collected. miR-600 expression was decreased in CRC tissue compared with adjacent normal tissue using qRT-PCR. **b** miR-600 expression in CRC cell lines (HCT116, SW480, HT29, LOVO, SW620) was significantly decreased compared with the normal human colon epithelial cell line NCM460, which was the lowest in SW620 cell line and highest in HCT116 cell line. **c** Compared with non-metastasis CRC tissue, miR-600 expression was decreased in metastasis CRC tissue. **d** Kaplan-Meier curve revealed a poor clinical prognosis for patients with low miR-600 expression. According to the average value of miR-600 expression, patients were divided into low miR-600 expression group (*n* = 47) and high miR-600 expression group (*n* = 29)

**Table 1:** Relationship between miR-600 expression and clinicopathological characteristics in colorectal cancer patients

Characteristics	Number	miR-600 expression		*P* value
		Low(*n* = 47)	High(*n* = 29)	
Age				0.690
≤ 60	31	20	11	
> 60	45	27	18	
Gender				0.677
Male	39	25	14	
Female	37	22	15	
Tumor location				0.284
Colon	40	27	13	
Rectum	36	20	16	
Tumor invasion depth				< 0.001*
T1, T2	24	6	18	
T3, T4	52	41	11	
Lymph node metastasis				0.022*
Yes	44	32	12	
No	32	15	17	
Distant metastasis				0.422
M1	11	8	3	
M0	65	39	26	

*Statistically signifcant

Next, we transfected miR-600 mimic or miR-600 inhibitor into SW480 and LOVO cell lines to overexpress or inhibit miR-600 (Fig. 2a), and evaluate the effects on cellular behaviors. Colony formation assay showed that the numbers of colonies were significantly decreased in miR-600-overexpressed SW620 and LOVO cell lines, whereas the numbers of colonies were increased in miR-600-inhibited HCT116 cell line (Fig. 2b). Wound healing assay showed that overexpression of miR-600 suppressed migration of SW620 and LOVO cells, and inhibition of miR-600 accelerated migration of HCT116 cells (Fig. 2c). Transwell assay showed that overexpression of miR-600 suppressed migration and invasion of SW620 and LOVO cells, and inhibition of miR-600 accelerated migration and invasion of HCT116 cells (Fig. 2d and e).

**Fig. 2:** miR-600 suppressed migration and invasion of CRC cells. **a** miR-600 mimic was transfected into SW480 and LOVO cell lines to overexpress miR-600, and miR-600 inhibitor was transfected into HCT116 cell line to inhibit miR-600 expression. **b** Colony formation assay showed that the numbers of colonies were decreased in miR-600-overexpressed SW620 and LOVO cell lines, and the numbers of colonies were increased in miR-600-inhibited HCT116 cell line. **c** Wound healing assay showed that overexpression of miR-600 suppressed migration of SW620 and LOVO cells, and inhibition of miR-600 accelerated migration of HCT116 cells. **d** Transwell assay showed that overexpression of miR-600 suppressed migration of SW620 and LOVO cells, and inhibition of miR-600 accelerated migration of HCT116 cells. **e** Transwell assay showed that overexpression of miR-600 suppressed invasion of SW620 and LOVO cells, and inhibition of miR-600 accelerated invasion of HCT116 cells

qRT-PCR analysis showed that overexpression of miR-600 suppressed N-cadherin, vimentin and Fibronectin expressions, and accelerated E-cadherin expression in SW620 and LOVO cells. Inhibition of miR-600 accelerated N-cadherin, vimentin and Fibronectin expressions, and suppressed E-cadherin expression (Fig. 3a). These findings proved miR-600 suppressed EMT in CRC cells. The findings of western blot analysis of the effect of miR-600 on E-cadherin, N-cadherin, vimentin and Fibronectin expressions were consistent with the findings of qRT-PCR (Fig. 3b). We transfected lenti-miR-600 or lenti-vector into SW620 cells, and established CRC xenografts in nude mice with lenti-miR-600 overexpression. miR-600 expression was significantly increased in lenti-miR-600 group, and overexpression of miR-600 significantly suppressed tumor volume and weight (Fig. 3c). Nude mice liver metastasis model of CRC was established to observe tumor nodules in liver tissues. We found overexpression of miR-600 significantly decreased the number of CRC liver metastasis after spleen injection (Fig. 3d).

RETRACTED

**Fig. 3:** miR-600 suppressed EMT related proteins in CRC cells and inhibited CRC growth in vivo. **a** qRT-PCR showed miR-600 suppressed EMT in CRC cells. Overexpression of miR-600 suppressed N-cadherin, vimentin and Fibronectin expressions, and accelerated E-cadherin expression in SW620 and LOVO cells. Inhibition of miR-600 accelerated N-cadherin, vimentin and Fibronectin expressions, and suppressed E-cadherin expression. **b** Western blot analysis of the effect of miR-600 on E-cadherin, N-cadherin, vimentin and Fibronectin expressions. **c** SW620 cells (transfected with lenti-miR-600 or lenti-vector) were subcutaneously injected into each BALB/c nude mice at a concentration of 1 × 10^6^ cells/100 μl (*n* = 6). Seven days after inoculation, tumor volume was measured. Nude mice were sacrificed after 25 days, then tumor tissues were weighed. miR-600 expression was increased in lenti-miR-600 group, and overexpression of miR-600 significantly suppressed tumor volume and weight. **d** SW620 cells (transfected with lenti-miR-600 or lenti-vector) were injected into the spleen subcapsular of each BALB/c nude mice at a concentration of 1 × 10^6^ cells/100 μl (*n* = 6) to establish nude mice liver metastasis model of CRC. Nude mice were sacrificed after 5 weeks, and liver tissues were obtained to count tumor nodules. Overexpression of miR-600 significantly decreased the number of metastatic nodules after spleen injection

RETRACTED

### KIAA1199 was upregulated in CRC cells

Using bioinformatics softwares (Targetscan and DIANA), the following potential targets of miR-600 that related to CRC migration were predicted, namely FOXG1, KIAA1199, IGF1R, MAP2K4, SCARA5, EFEMP1, IRS1, RAB22A, RAB1A, ATF3, HMGB1. The expressions of these genes in CRC tissues and adjacent normal tissue were downloaded from Gene Expression Omnibus (GEO, GSE21510), which found the expression of KIAA1199 in CRC tissue was significantly higher than normal tissue (Fig. 4a). qRT-PCR analysis also showed that KIAA1199 mRNA level was upregulated in CRC tissues than adjacent normal tissues (Fig. 4b).

**Fig. 4:** miR-600 suppressed KIAA1199 expression and inhibition of KIAA1199 suppressed migration and invasion of CRC cells. **a** Target proteins related to CRC migration (FOXG1, KIAA1199, IGF1R, MAP2K4, SCARA5, EFEMP1, IRS1, RAB22A, RAB1A, ATF3, HMGB1) were screened in genes having binding sites with miR-600 predicted by bioinformatics software (Targetscan and DIANA). The gene expressions in CRC tissues and adjacent normal tissue were downloaded from GSE21510 in Gene Expression Omnibus (GEO). The expression of KIAA1199 in CRC tissue was significantly higher than normal tissue. **b** qRT-PCR was performed to measure mRNA level of KIAA1199 in 76 CRC tissues and adjacent normal tissues. Compared with adjacent normal tissues, KIAA1199 mRNA level was upregulated in CRC tissues. **c** Binding sites between miR-600 and KIAA1199. SW620 cells were transfected with miR-600 mimic or pre-NC. miR-600 mimic significantly decreased luciferase activity of KIAA1199 WT, and there was no significant difference in the activity of KIAA1199 MUT. HCT116 cells were transfected with miR-600 inhibitor or NC. miR-600 inhibitor significantly increased luciferase activity of KIAA1199 WT, and there was no significant difference in the activity of KIAA1199 MUT. **d** miR-600 mimic significantly decreased KIAA1199 expression in SW620 and LOVO cells, whereas miR-600 inhibitor significantly increased KIAA1199 expression in HCT116 cells. **e** si-KIAA1199 significantly suppressed KIAA1199 expression in SW620 and LOVO cells. **f** Wound healing assay showed that si-KIAA1199 suppressed migration of SW620 and LOVO cells. **g** Transwell assay showed that si-KIAA1199 suppressed migration and invasion of SW620 and LOVO cells

Luciferase reporter method was used to detect whether miR-600 can directly target KIAA1199 3’UTR. KIAA1199 WT sequence or KIAA1199 MUT sequence were cloned into the luciferase reporter vector. Then, KIAA1199 WT or MUT and miR-600 mimic or inhibitor were transfected into SW620 or HCT116 cells. We observed a significantly decrease in the luciferase activity of KIAA1199 WT vector after transfected with miR-600 mimic in SW620 cells, and there was no significant difference in the activity of KIAA1199 MUT (Fig. 3c). We observed a significantly increase in the luciferase activity of KIAA1199 WT vector after transfected with miR-600 inhibitor in HCT116 cells, and there was no significant difference in the activity of KIAA1199 MUT (Fig. 3c), providing the evidence of direct interaction between miR-600 and KIAA1199. miR-600 mimic significantly decreased KIAA1199 expression in SW620 and LOVO cells, whereas miR-600 inhibitor significantly increased KIAA1199 expression in HCT116 cells (Fig. 4d), which indicated that KIAA1199 was negatively regulated by miR-600.

RETRACTED

### KIAA1199 promoted CRC cell migration and EMT

As shown in Fig. 4e, si-KIAA1199 significantly suppressed KIAA1199 expression in SW620 and LOVO cells. What’s more, wound healing assay (Fig. 4f) and Transwell assay (Fig. 4g) showed that si-KIAA1199 suppressed migration and invasion of SW620 and LOVO cells, whereas KIAA1199 overexpression promoted CRC cell migration and invasion, which rescued the inhibition effect of miR-600 mimic on migration and invasion of CRC cells (Fig. 5a and b). Western blot analysis showed that KIAA1199 overexpression promoted EMT related proteins, which rescued the inhibition effect of miR-600 mimic on the expression of N-cadherin, vimentin and Fibronectin (Fig. 5c).

**Fig. 5:** KIAA1199 overexpression reversed the inhibition effect of miR-600 mimic on migration and invasion of CRC cells. SW620 and LOVO cells were transfected with NC, miR-600 mimic, miR-600 mimic+pcDNA, miR-600 mimic+pcDNA-KIAA1199. **a** Transwell assay showed that KIAA1199 overexpression reversed the inhibition effect of miR-600 mimic on migration of CRC cells. **b** Transwell assay showed that KIAA1199 overexpression reversed the inhibition effect of miR-600 mimic on invasion of CRC cells. **c** Western blot analysis showed that KIAA1199 overexpression reversed the inhibition effect of miR-600 mimic on the expression of N-cadherin, vimentin and Fibronectin, and the promotion effect of miR-600 mimic on the expression of E-cadherin

### LncRNA TUG1 negatively regulated miR-600 to accelerate cell metastasis and EMT in CRC

According to the prediction result of bioinformatics software (DIANA), there were binding sites between TUG1 and miR-600. TUG1 WT or TUG1 Mutant sequences were cloned into the luciferase reporter vector. Then, TUG1 WT or TUG1 MUT and miR-600 mimic or pre-NC were transfected into SW620 cells. We observed a significantly decrease in the luciferase activity of TUG1 WT after transfected with miR-600 mimic, and there was no significant change in the activity of TUG1 MUT, indicating miR-600 directly bound to TUG1 (Fig. 6a). qRT-PCR analysis showed that si-TUG1 significantly decreased TUG1 level and increased miR-600 level in SW620 and LOVO cells (Fig. 6b), whereas pcDNA-TUG1 significantly increased TUG1 level and decreased miR-600 level in HCT116 cells (Fig. 6c). Then, Ago2 antibody was added into SW620 cell lysate for RIP. qRT-PCR showed that TUG1 and miR-600 enrichment was significantly increased in Ago2 than IgG (Fig. 6d). We also observed TUG1 level was negatively correlated with miR-600 level in CRC tissue (Fig. 6e). Transwell assay (Fig. 6f) and Western blot analysis (Fig. 6g) showed that miR-600 inhibitor rescued the inhibition effect of si-TUG1 on the migration/ invasion of CRC cells and EMT related protein expression.

RETRACTED

**Fig. 6:** TUG1 regulated miR-600 expression and influence the effect of miR-600 on the migration of CRC cells. Bioinformatics software (DIANA) predicted binding sites between TUG1 and miR-600. **a** Binding sites between TUG1 and miR-600. Luciferase reporter gene vector containing TUG1 WT or TUG1 Mutant were co-transfected with miR-600 mimic or pre-NC into SW620 cells. Dual-luciferase reporter gene assay showed that miR-600 mimic significantly decreased luciferase activity of TUG1 WT, and there was no significant change in the activity of TUG1 Mutant, indicating miR-600 can bind with TUG1. **b** qRT-PCR showed that si-TUG1 significantly decreased TUG1 level and increased miR-600 level in SW620 and LOVO cells. **c** pcDNA-TUG1 significantly increased TUG1 level and decreased miR-600 level in HCT116 cells. **d** Ago2 antibody was added into SW620 cell lysate for RIP. qRT-PCR showed that TUG1 and miR-600 enrichment was significantly increased in Ago2 than IgG. **e** TUG1 level was negatively correlated with miR-600 level in CRC tissue. **f-g** SW620 cells were transfected with si-NC, si-TUG1, si-TUG1 + NC, si-TUG1 + miR-600 inhibitor. Transwell assay showed that miR-600 inhibitor reversed the inhibition effect of si-TUG1 on the migration and invasion of CRC cells. Western blot analysis showed that miR-600 inhibitor reversed the effect of TUG1 on EMT related protein expression

## Discussion

Numerous studies have shown that lncRNAs play critical role in modulating tumor processes, such as apoptosis, proliferation and metastasis [20, 21]. Although our previous report has proved lncRNA TUG1 promoted the aggressiveness of CRC cells and facilitated EMT in CRC cells [19], the exact molecular mechanism mediated by lncRNA TUG1 in CRC is still unclear. So, we further attempted to reveal the possible mechanism of lncRNA TUG1 mediated CRC metastasis in this study. It has been reported that lncRNAs could facilitate or suppress tumor processes via competitively binding with miRNAs, and bioinformatics software analysis is commonly used to predict the potential binding sites between miRNA and the interacted genes [22]. In this study, bioinformatics software DIANA predicted there were potential binding sites between TUG1 and miR-600. We observed TUG1 knockdown increased miR-600 expression in CRC cells, whereas overexpression of TUG1 decreased miR-600 expression. Besides, TUG1 knockdown suppressed CRC cell migration and invasion and EMT, and miR-600 inhibitor reversed these inhibition effects, indicating lncRNA TUG1 could negatively regulated miR-600 to promote migration and invasion of CRC cells and EMT in CRC cells.

RETRACTED

Evidence has shown that miRNAs play critical roles in modulating proliferation, metastasis and EMT of CRC, such as miR-590-5p, miR-198, miR-19b-3p, etc. [23–25]. miR-600 is a newly identified miRNA and its role in proliferation, apoptosis, migration in cancer cells is largely unknown. Zeng et al. reported that miR-600 could be significantly associated with prolonged survival time in cervical cancer [17]. Zhang et al. found that miR-600, as a negative regulator of p53, could suppress proliferation, migration and invasion in mutant p53-expressing human CRC cell [18]. However, the expression of miR-600 in CRC cell lines or tissues has not been discussed, and its role in EMT and CRC metastasis has not been explored. In this study, we focused on the role of miR-600 in migration and invasion of CRC cell, EMT in CRC cells and CRC metastasis. We observed that miR-600 was downregulated in CRC tissues and cell lines and CRC metastatic tissue, and low miR-600 expression predicted a poor clinical prognosis for CRC patients. Besides, we found overexpression of miR-600 inhibited migration and invasion of CRC cells, which was consistent with previous report [18]. Moreover, miR-600 overexpression inhibited EMT in CRC cells in vitro, suppressed tumor volume and weight in vivo, and reduced the number of liver metastasis in vivo, which brought new evidence to the role of miR-600 in CRC progression.

KIAA1199, also defined as cell migration inducing protein (CEMIP), has been reported to be overexpressed in many cancers and promoted cancer metastasis through different signaling pathways, such as Wnt signaling and MEK1/ERK1/2 signalling [26, 27]. Evensen et al. found KIAA1199 was upregulated in breast cancer metastatic tissues, and resulted in EMT in breast cancer cells, inhibited cell migration in vitro and decreased metastasis in vivo [8]. Recently, researchers showed that KIAA1199, one of the direct targets of miR-216a, was highly expressed in CRC metastatic tissues, and KIAA1199 downregulation inhibited CRC cell migration and invasion in vitro [12]. However, there was no research studying the function of miR-600 on KIAA1199 in CRC metastasis. Our present study first proved that KIAA1199 was a direct target of miR-600, and was negatively regulated by miR-600 to modulate CRC cell migration and invasion, revealing new mechanism of miR-600 on CRC progression.

RETRACTED

### Limitations

our study had a relatively small sample size which may be an important factor affecting the extrapolation of our results. The statistical test for miR-600-related survival is of borderline significance. Thus, a larger study should be performed to clearly determine the relationship between miR-600 expression and CRC patients survival.

## Conclusion

In this study, we discovered miR-600 was downregulated and KIAA1199 was upregulated in CRC tissues and cell lines, which predicted a poor clinical prognosis. Overexpression of miR-600 suppressed CRC cell migration/invasion and EMT-related proteins, inhibited tumor volume and weight, and decreased the number of CRC liver metastasis via KIAA1199. Inhibition of TUG1 suppressed CRC cell migration and invasion and EMT-related proteins via regulating miR-600. Our study first proved that TUG1/miR-600/KIAA1199 promoted CRC cell migration and EMT in vitro and metastasis in vivo.
